The article "Modeling Hypertension as a Contributor to Retinal Hemorrhaging from Abusive Head Trauma" was published in 2020. Journal: J Healthc Eng.

# Modeling Hypertension as a Contributor to Retinal Hemorrhaging from Abusive Head Trauma

**DOI:** 10.1155/2020/4714927

**Published:** 2020-05-20

**Authors:** Christopher Umstead, Alan Barhorst, Thivakorn Kasemsri, Kelly Mitchell

**Affiliations:** ^1^Texas Tech University, Department of Mechanical Engineering, Box 41021, Lubbock, TX 79430-9406, USA; ^2^Texas Tech University Health Sciences Center, Department of Pediatrics, Division of Pediatric Critical Care, 3601 4th Street, Lubbock, TX 79430-9406, USA; ^3^Texas Tech University Health Sciences Center, Department of Ophthalmology & Visual Sciences, 3601 4th Street, Lubbock, TX 79430-9406, USA

## Abstract

Retinal hemorrhaging (RH) is indicative and prevalent in abusive head trauma (AHT)—yet the direct cause of the RH from AHT is unknown. Our hypothesis is that RH in AHT is the combination of shaking forces and hypertension. This combination of effects explains why RH is not normally observed in common childhood accidents but is nearly exclusively observed in AHT. An experimental model using porcine eyes was designed to ascertain the required pressure change for sudden RH and, via a computer model, the subsequent stress increase in blood vessels. The porcine eyes were cannulated via the maxillary artery and pressurized until perfusion and RH were observed. Fluid was injected into the head with a computer-controlled continuous flow syringe pump; video of the fundus was recorded during perfusion; and the pressure of the fluid entering the eye was recorded as well. A computer model was created in COMSOL to simulate loading from hypertension, shaking, and the combination of the forces. This model was validated via experimental data collected from the porcine model. It was found that hypertension or shaking alone did not cause an increase in stress required to cause RH. But when the loading of shaking and hypertension was combined, as would occur in AHT, the stress increases were greater than those extrapolated from the porcine model and would cause RH.

## 1. Introduction and Review

Abusive head trauma (AHT) is an affliction committed upon the defenseless with no externally visible trauma but lasting brain injuries. AHT, also known as shaken baby syndrome, occurs when a caretaker grabs the infant by the trunk and violently shakes the infant; the motion of the head whipping back and forth causes brain and eye hemorrhaging [1]. The two prevailing theories of the mechanism of traumatic brain injury (TBI) in AHT are as follows: the brain contacts the skull causing bruising and concussions, and the blood vessels between the dura and pia mater are torn by the movement of the brain in the skull [2, 3]. Neither of the injury mechanisms requires external impacts to the head, but determining if abuse has occurred without reasonable doubt has proven problematic. Approximately 1400 infants each year suffer from this abuse with a fatality rate of approximately 30% [4]. The only visible indication that AHT has occurred is retinal hemorrhaging (RH) [5]. RH occurs in upwards of 85% of confirmed cases of AHT [6–8]. Damage to the eye may require more trauma than needed to inflict harm to the brain—implying if RHs are present, then most likely subdural hemorrhaging has occurred [9]. But the mechanism of RH from AHT is unproven. We propose that hemorrhaging occurs from a combination of shaking forces and an increase in blood pressure due to hypertension [10].

The article "Modeling Hypertension as a Contributor to Retinal Hemorrhaging from Abusive Head Trauma" was published in 2020. Journal: J Healthc Eng.

Retinal hemorrhaging is prevalent in TBI from AHT, and the severity of the brain injury positively correlates with the extent of RH [6, 11–13]. RH was observed in 80% of AHT cases documented, while RH was only observed in less than 12% of the accidental TBI [6, 11–13]. RH can appear in the shape of a dot or a flame and both types of hemorrhages are visible in AHT and were observed in our porcine model [14, 15]. Over a third of the AHT cases had no external indications of injuries [11, 13]. In both accidental and inflicted TBI, spinal injury was absent [13]. Differentiating accidental TBI from AHT is the presence of external injures such as bruises, bone fractures, and skull fractures; moreover, the external injuries observed on the infants are consistent with accidents and the testimonies of the witnesses and caretakers [11, 13]. The most devastating injury from AHT is damage to the brain.

The engineering community has postulated that strains and stress in the eye from shaking can cause the blood vessels to rupture [16–18]. Finite element models have concluded that abuse could subject the eye to enough force to cause RH. Anthropomorphic models have been used to ascertain acceleration force from shaking, falling, and other activities, both benign and malevolent, as applied to infants. Adult volunteers violently shook anthropomorphic dolls to simulate AHT; the volunteers were able to produce angular accelerations upwards of 1068.3 rad/s^2^ [19–22]. The measured acceleration from abuse was substantially more than that from normal activities but less than the required acceleration to cause brain damage from a single dropping event. The angular velocity profile from Prange's experiment is used in this paper's computer model of RH [19].

One of the responses of the body to trauma is hypertension, that is, blood flow and pressure are increased to provide aid to the injured organ. Hypertension increases the stress load in the blood vessel walls as shown in the computer model. In children (0 years to 15 years) with blunt trauma, the systolic blood pressure substantially increased above the norm [23, 24]. The heart rate increases a little in injured children but not significantly when compared to the heart rate of healthy children. For infants (<1 year), the average systolic blood pressure for blunt injury was 105 mmHg which is an increase of 14 mmHg above the norm [23]. The increase in systolic blood pressure for TBI cases was similar to the pressure increase in blunt injuries. Infants with TBI had an average blood pressure of 117 mmHg which is an increase of 26 mmHg above the norm [24]. The arterial blood pressure in the CRA (central retinal artery) is directly related to the systolic pressure, so an increase in the systolic pressure will also increase the blood pressure in the CRA [25].

The article "Modeling Hypertension as a Contributor to Retinal Hemorrhaging from Abusive Head Trauma" was published in 2020. Journal: J Healthc Eng.

Blood pressure is the greatest when it leaves the aorta and decreases as the blood circulates throughout the body. The pulsating pressure wave in the blood, created by the heart pumping, is damped by the elastic properties of the arteries, so the blood pressure is considered to be constant in the smaller arteries [26]. The blood pressure of the ophthalmic artery directly corresponds to the brachial artery pressures at a ratio of 0.68 [27]. The volumetric flow rate of the blood is proportional to the diameters of these blood vessels in healthy subjects. The vessels are between 72 and 185 *µ*m in diameter for an eye in an adult male; the volumetric flow is between 38.1 ± 6.2 and 43.4 ± 8.9 *µ*l/min and the correspond flow rate was found for the model section [28]. The blood leaves the eye at a venous pressure between 15 and 20 mmHg, which is slightly higher than the intraocular pressure [29]. From the above, the blood pressure in the ophthalmic artery in AHT cases would range from 57 mmHg to 79.6 mmHg.

Sufficiently high blood pressure within the eye globe has been shown to cause RH, and some have postulated that hypertension can cause RH in AHT [13, 14, 30, 31]. Yet the contrary evidence for increased resistance in the vein as a cause of RH from AHT is the observation that central retinal vein obstruction produces RH with distinguishable patterns that are not observed in AHT [6, 7]. Yet the direct pressure necessary to facilitate immediate RH has not been determined either experimentally or empirically.

RH has been observed in bungee jumpers, while bungee jumping is an adult activity; the physical forces on the eye and physiological responses in the body from bungee jumping are similar to AHT. The physicians tending to the bungee jumping cases attributed the RH to the rapid deacceleration and increased pressure in the eye circulatory system [32, 33]. So RH from bungee jumping supports the hypothesis that hemorrhaging can be produced from a combination of acceleration and hypertension without physical contact.

The article "Modeling Hypertension as a Contributor to Retinal Hemorrhaging from Abusive Head Trauma" was published in 2020. Journal: J Healthc Eng.

Porcine eyes were selected for the experiment due to the similarities of brain morphology and anatomy to humans [34]. RH has been examined in pigs subjected to rapid acceleration and impacts to the head; however, the results have been ambiguous. Young piglets subjected to a single rapid axial rotation did not exhibit any RH [35]. Yet, in a very similar experiment, 73% of piglets subjected to rapid transverse rotation exhibited RH [36]. The path of blood flow to and from a porcine eye is summarized in Figure 1. Because the eye shares the same source of blood as the face, the blood flow is subjected to disruption during other bodily activities [37–39]. Within the globe, both porcine eyes and human eyes exhibit holangiotic properties that are similar, but there are some differences within the capillaries and construction of the layers of the eye. The major vessels within the human retina reside deeper compared to the porcine eye which are close to the limiting membrane and protrude into the vitreous. The porcine and infant eyes share the important characteristics of the capillaries of net distribution, and the porcine capillaries are slightly less in depth in the retina [37]. These characteristics make the isolated porcine eye viable for experiments simulating forces and loads on the retina in lieu of using human eyes.

## 2. Porcine Ex Vivo Hypertensive Experiment

To simulate hypertension in the eye, an ex vivo model was developed. Porcine eyes were cannulated, and fluid was perfused throughout the eye. The pressure of the fluid was increased until RH was observed via an endoscope inserted through the limbus. The fluid pressure and flow rate were controlled and recorded along with video of the fundus via a computer interface for postanalysis. Details of the model as described in the overview are given below.

### 2.1. Materials and Methods

Porcine heads were obtained from a Texas Tech Dept. of Animal and Food Sciences nutrition research project [40]. The pigs were from the Iowa State University RFI herd, about 6 months old, and weighed approximately 70 kg at the time of sacrifice. The animals were euthanized with Fatal-Plus per the department's protocols. The heads were separated from the body at the C1 vertebrae and stored on ice. All the animals were utilized within 40 hours of death with an average delay of 19 hours.

Cannulation of the eye was accomplished via the maxillary artery. An 8 by 10 cm window was created just inferior of the eyelid in the head. Any visible muscle, specifically the masseter, was removed. The zygomatic arch was cut near the edge of the window and removed along with any newly exposed flesh. The exposed mandible was removed. The ophthalmic artery and vein, which are located near the sphenoid bone under the flesh beneath the mandible, were exposed. A small slit was made in the maxillary artery. Silastic tubing (2.41 mm OD, 1.57 mm ID) was inserted into the artery, pushed to the base of the eye, and secured in place with sutures [10].

The article "Modeling Hypertension as a Contributor to Retinal Hemorrhaging from Abusive Head Trauma" was published in 2020. Journal: J Healthc Eng.

A syringe pump, pressure transducer, borescope, and camera in conjunction with a computer interface were arranged as depicted in Figure 2 and used to inject fluid into the eye while recording video of the fundus. A continuous flow syringe pump (Harvard PHD HA 2000 Push-Pull/Continuous Flow Configuration, INSTECH, Plymouth Meeting, PA) was used to inject Krebs-Ringer Bicarbonate solution with green fluorescein salt into the eye. The flow rate of the injection was controlled with a custom interface created in LabVIEW (National Instruments, Austin, Texas). A pressure transducer (PX309, Omega Engineering Inc., Stamford CT) was situated to record the pressure of the flow just before the fluid entered the head. A small slit was made in the lens of the eye through which a borescope with an attached camera (1800 Endoscope, Bradenton FL) was inserted into the globe; video of the fundus was compressed and recorded in LabVIEW.

Perfusion of the eye was confirmed by observation of dye in the arteries of the retina as shown in Figure 3. The eyes were rejected if no dye was observed in the fundus. The pressure and the flow were recorded at all times during the experiment while the video recording was selectively activated to conserve computer memory. A correction factor was applied to the data to account for the pressure lost between the transducer and point of cannulation. The correction factor was determined by cutting the tube proximally as possible to the eye and recording the pressure for flow rates in the open tubes.

### 2.2. Results

The results of the experiment were analyzed in Microsoft Excel 2007 (Microsoft, Redmond, WA) and in Minitab 17 (Minitab, State College, PA). An alpha confidence level of 0.05 was used for all statistical tests. Normality was observed in perfusion pressure (*p*=0.12), settling pressure (*p*=0.07), choroid perfusion (*p*=0.27), and RH pressure (*p*=0.97). Variance was similar across all groups (*p* > 0.05). One-tailed *t*-tests were used to compare the settling pressures with retinal perfusion pressures and RH pressures.

Perfusion of the eye was observed in 17 eyes in 11 of the swine heads. The green Krebs solution was observed to perfuse throughout the retina as shown in Figure 3. The pump overcame the resistance of clotted blood at an average pressure of 39.89 mmHg (SD = 15.73) at a flow rate of 100 *μ*l/min (mode, *n* = 11). The pressure dropped after overcoming the initial resistance to an average steady pressure (*M* = 28.61 mmHg, SD = 15.40, *t* = 2.00, *p*=0.027). Perfusion of choroid occurred in 8 of the eyes observed as a dull green staining superficial to the retina at an average pressure of 32.14 mmHg (SD = 14.11).

The article "Modeling Hypertension as a Contributor to Retinal Hemorrhaging from Abusive Head Trauma" was published in 2020. Journal: J Healthc Eng.

As the pressure increased in the eye, RH was observed as bright green spots—normally appearing near bifurcations of the artery as shown in Figure 4. RH was first observed at an average pressure of 39.45 mmHg (SD = 11.43). The pressure to facilitate rupture was greater than the settling pressure with a mean difference of 10.84 mmHg (*t* = 2.01, *p*=0.028). The number of ruptures increased, as can be observed in Figure 5, as time passed and pressure increased in the eye in a similar pattern as observed in AHT.

## 3. AHT Computer Model

To calculate the stress increase from shaking and hypertension both isolated and combined, a computer model was created in COMSOL Multiphysics (v4.4, Burlington, MA). The same model was created from a picture from the animal experiment. Five primary models were created to compute the stress in the retina: models using the pressure and flow results from the porcine experiments; a control model using the blood pressure from a healthy infant; a model using hypertension for TBI; a model using simulating shaking alone; and a model that combines both the shaking and hypertension. The stress location and increase were validated and compared against the results from the animal experiments.

The fundus image was selected for importation into the computational model because RH was visible allowing for comparison between the finite element analyses (FEAs) and the experimental model results. Because hemorrhaging of the vessels was observed to leak into the retina and not into the vitreous humor or between the retina and choroid layer, the computer model utilized a thin 2D section of the retina for analysis. The image was first imported into the drafting software from DraftSight (V1R4, Dassault Systemes, Velizy-Villacoublay, France). The edge of blood vessels in the fundus was manually traced as shown in Figure 6, creating 9 distinct domains for the tissue of the retina (r), the blood vessel walls (w), and the blood (b). The domain files were imported in COMSOL Multiphysics and scaled to human eye proportions. The COMSOL package for fluid-structure Interaction (fsi) was used to compute the displacement and stress within the fundus due to hypertension. To compare the simulation results from all the loading conditions, 4 points of interest (POI) were selected at the center of the model near the bifurcations and bends.

The article "Modeling Hypertension as a Contributor to Retinal Hemorrhaging from Abusive Head Trauma" was published in 2020. Journal: J Healthc Eng.

### 3.1. Eye Material Properties

The material properties for the tissues of the retina, artery walls, and blood have been described in the literature and are given in Table 1 [41–44]. In a few cases, the material properties were not located for human tissue and the values for either bovine or porcine tissue properties were substituted. The bovine retina density was used for the retina material [41]. The porcine Poisson's ratio and Young's modulus were used for the blood vessel walls in the model [44]. The dynamic viscosity of the blood was determined using Ramplings' data and is given in the following equation [45]: where *μ* is the viscosity and $\dot{\gamma }$ is the shear rate.

(1) $$\begin{array}{c} \mu =28.52*{\dot{\gamma }}^{-0.385}, \end{array}$$

### 3.2. Blood Velocity Outlet

The outlet conditions were held constant across all infant models. The normal flow velocity of the blood was determined by interpolating the values from Grunwald's paper [28]. The length of each outlet was measured, and the corresponding exit velocity and the flow rate for outlet o1, o2, and o3 are given in Table 2. The outlet was assumed to be cylindrical in shape, so the normal velocity and velocity profile were computed by COMSOL.

### 3.3. Blood Pressure Input

 the normal blood pressure from a healthy infant and the pressure increase from hypertension due to TBI. An ophthalmic artery blood pressure of 63 mmHg for a healthy 6-month-old infant, as described above, was used for the baseline model. The afflicted hypertension for the ophthalmic artery pressures of 79.6 mmHg was used for the TBI and AHT computer models.

### 3.4. Abusive Acceleration

From anthropomorphic models, Prange et al. were able to measure the angular velocity of the head from simulated abusive shaking [19]. From the angular velocity, the normal acceleration was computed and converted to a body load for each element using equation (2) where *F* is the force, *ρ* is the density, *r* is the distance from the chest to the eye, and *ω* is the angular velocity. The computed loads were applied to both the solid and fluid domains in the FEA model in the direction to cause the greatest stress increase in the vessels:

(2) $$\begin{array}{c} F_{\text{body}}=\rho *r*\text{sign}\left(\omega \right)*\omega^{2}. \end{array}$$

### 3.5. Computer Model Validation

The location of the stress and strain concentration in the FEA model and the RH in the porcine model had a positive spatial correlation. As can be observed in Figure 7, the locations of the strain, in the same location of the stress concentrations, occurred in the same area as the hemorrhaging observed in the porcine retina which are indicated with the arrows. This correlation gives credence to the spatial accuracy of the FEA model. The spatial validation supports the computation of, although not directly measure, the increase of stress predicted by the FEA model.

The article "Modeling Hypertension as a Contributor to Retinal Hemorrhaging from Abusive Head Trauma" was published in 2020. Journal: J Healthc Eng.

### 3.6. Ex Vivo RH Experimental Model

The results from the porcine experiments were used to build a baseline FEA model and establish the stress increase to facilitate RH. The flow rate into the eye used in the experiment was divided by six to account for the number of arteries entering the fundus and applied at the inlet of the FEA model. The pressure drop across the model domain was negligible, so measured pressure was applied to each of the outlets in the model to satisfy computation requirements. The change in stress required to cause RH was determined by finding the difference between the settling pressure and the observed RH pressure. The settling pressure had an inlet flow velocity of 2.46 cm/s and a pressure of 28.61 mmHg was applied to the outlets. The von Mises stress values for the POIs are given in Table 3 along with the displacements and volumetric strain. The observed RH pressure model had an average flow velocity of 14.73 cm/s which was 50% more than the observed settling pressure model; a pressure of 39.46 mmHg was used at the fluid exits which was an increase of 38% above the settling pressure outlets. The von Mises stress values for the POIs are given in Table 4, and they had an average increase of 40% over the settling pressure. The RH model POI displacements were 48% more than the settling model.

### 3.7. Healthy Infant Baseline Model

A baseline control model was made using the parameters of a healthy six-month-old infant. A blood pressure of 63 mmHg was used to compute the initial internal stress in the retina. The computed fluid pressure drops by 1.6 mmHg from the inlet compared to the outlet, and this is a reduction of 1.6%. The initial displacement of the tissue was also determined for reference. The von Mises stress values for the points of interest are presented in Table 5 along with the displacements.

### 3.8. TBI Infant Models

The TBI best simulates the stress in the eye from hypertension alone due to abuse. Using Loizou's injury data, the hypertensive ophthalmic blood pressure was calculated to be 79.6 mmHg for injured infants with TBI [24]. The von Mises stress within the artery walls was near 7000 Pa, which was a 30% increase over the baseline wall stress. The von Mises stress in the center of the retina was between 500 Pa and 1000 Pa. The von Mises stress values of the POIs in Table 6 are on average 20% above the baseline model. The displacements were 34% more for the POIs than in the healthy infant. The maximum displacement was 19% greater than that of the healthy infant model and occurred at the same location as the other models.

The article "Modeling Hypertension as a Contributor to Retinal Hemorrhaging from Abusive Head Trauma" was published in 2020. Journal: J Healthc Eng.

As expected, the increase of the stresses in the eye had a strong correlation with the increases in blood pressure. The results for the POI stresses as a function of the blood pressure are discussed below. The linear relationship was very strong (*r*^2^ ≈ 0.99) for the average von Mises stress as a function of blood pressure. For a change in pressure, the stress increased the most for the TBI infant models with the greatest numerical increase of 283 Pa at POI4 and the greatest percentage increase of 28% occurred at POI2 as compared to the healthy infant eye. The least numerical increase in the von Mises stress compared to the baseline model was 29.1 Pa which occurred at POI1. The von Mises stress increased by the least of 2.9% at POI3. The preliminary results establish that the model was behaving as expected and properly constrained. The stress increase from hypertension alone was not significant enough to cause failure when compared to the failure stress increase in the porcine model. The maximum displacement occurred in the same location for all models near POI3. The maximum displacement for the POI, like the other models, occurred for the TBI infant models, at POI3 which was 4.7 *µ*m more than the baseline model, which is an increase of 36%.

### 3.9. Abusive Shaking TBI Model

The body force from abusive shaking was applied to the AHT model along with the hypertensive ophthalmic blood pressure of 79.6 mmHg [24]. This model best simulates the stress in the eye from isolated hypertension due to the TBI from AHT. The average and maximum values of stress and displacement are given in Table 7. The maximum von Mises stress increased by 28% compared to the baseline model. The greatest percentage increase of 50% in the von Mises stress occurred for POI2 after 1 second of shaking. The greatest von Mises stress increase was 37% and 26% for POI1 and POI4, respectively, which also occurred simultaneously.

### 3.10. Sans Hypertensive Shaking Model

The shaking acceleration was also applied to a nonhypertensive model using a healthy blood pressure of 63 mmHg. The stress from shaking alone was less than the stress caused by hypertension. The maximum displacement of 17.7 *µ*m for the POIs occurred at POI3. The values for stress and displacement for remaining the POIs are given in Table 8.

The increase in stress from shaking acceleration alone was minimal compared to the TBI infant models. Compared to the TBI model, the average displacement increased by 24% for the acceleration field and the von Mises stress increased by an average of 12%. The maximum POI displacement difference for shaking compared to the TBI was 67% and occurred for POI4. While the average stress between the shaking model and the TBI model was similar, the maximum displacement and stress were significantly greater in the shaking model.

The article "Modeling Hypertension as a Contributor to Retinal Hemorrhaging from Abusive Head Trauma" was published in 2020. Journal: J Healthc Eng.

## 4. Correlation of Experimental Data and the Computation Study and Discussion

As mentioned, the spatial correlation between the porcine and the FEA model was strong. In Figure 7, the model is paired with the same section of the porcine model fundus from which it was created. In the figure, the stress concentration in the arteries in the FEA model can be seen in the left image paired with the corresponding RH in the porcine model fundus in the two right images. The initial RH, seen in the top image, continued to develop as the pressure was increased as can be observed in the lower right image. The porcine model arteries ruptured in the same locations as predicted by the FEA model, and the locations of the RH matched the location of the stress increase indicated by arrows in Figure 7.

The increase between the models and the baseline computer model is tabulated in Table 9. The increase in stress to cause RH in the porcine FEA model was an average of 39% for the von Mises stress. The computed maximum stress increase for the hypertensive models and steady-state abusive models was significantly less than the stress increase in the porcine model. The stress in the nonhypertensive model, subjected to shaking, was also less than the computer-based rupturing stress. The volumetric strain and displacement in the shaking simulation were greater than the strain required to cause RH in the porcine model.

When the section of the fundus in the FEA model was subjected to hypertension from traumatic brain injury (TBI), the increase in stress and strain was significantly less than the increase needed to cause RH. Nor was the stress increase enough to cause RH when the model was subjected to forces from shaking alone (sans hypertension). But in each case, the locations of the increased stresses corresponded with where RH was observed in the porcine model.

When the FEA model was subjected to both hypertension and the force from shaking, the stress increase was compounding. The stress and strains from the combined loading were greater than the computed increase from the baseline porcine FEA model. In several cases, as shown in italics in Table 9, the increase was significantly greater than that in the porcine model. Therefore, the model simulation supports the hypothesis that hypertension in combination with the forces from shaking is a contributor to RH in AHT.

The article "Modeling Hypertension as a Contributor to Retinal Hemorrhaging from Abusive Head Trauma" was published in 2020. Journal: J Healthc Eng.

The mechanism of RH due to hypertension is feasible given that pressure change is comparable to the pressure increase required to cause RH in the animal model. Additionally, the eyes are under stress from the sustained movement during abuse, and this along with the stress from hypertension provides a likely reason why RH occurs nearly exclusively in AHT. The forces and stresses in accidents are separated by time from hypertension which occurs after the injury. In AHT, the stresses from both acceleration and hypertension occur simultaneously causing RH.

The change in pressure required to cause the blood vessels to rupture is within the realm of change in blood pressure due to hypertension. Blunt trauma causes a rise in systolic pressure of 22 mmHg in infants [23, 24]. The pressure in the ophthalmic artery corresponds proportionally to the pressure in brachial artery pressure [25, 27]. So, the retina artery endures a substantial increase in blood pressure from hypertension caused by trauma. The porcine model demonstrates that RH can be caused by pressure alone. The porcine eyes only required an increase of 10.84 mmHg in pressure to cause RH which is less than the increase from hypertension infants; considering that the vasculature in the pig retina is shallow in comparison with humans, less pressure to facilitate rupture is expected [37]. Systemic malignant hypertension alone can cause RH which occurs days to weeks later after the onset of high blood pressure [13, 14, 30, 31]. But the stresses in the vessel would occur instantaneously from hypertension, which when compounded with the stress from being shaken can cause the vessels to break instantaneously. For that reason, a hypertensive increase in blood pressure should be considered to have a significant role in causing hemorrhaging in the eye from AHT.

The increase in stress to cause RH in the porcine FEA model presented was an average of 39% for the von Mises stress. The computed maximum stress increase for the hypertensive models was significantly less than the stress increase in the porcine model. The stress in the nonhypertensive model, subjected to shaking, was less than the computer-based rupturing stress. As observed in the FEA model, hypertension causes significant stress increase within the retina. Also stress from shaking san hypertension was less than the stress from hypertension alone. Neither condition independent of the other exceeded the computed stress increase in the porcine eye.

In AHT, the infant's eye will be subjected to both shaking and hypertensive stress. As the infant is being shaking, the body has an injury adaptive response and hypertension occurs. The combined stress from the two loading conditions, shaking and hypertension, exceeded the increase to cause RH in the baseline porcine model. The combination of stresses provides an explanation for why RH is not observed in common childhood accidents but is observed in AHT [10]. In a fall or similar common accidents, the stresses from the physical injury are isolated in time from the physiological response of the body because the duration of the injury event is short and the body response occurs after the injury mechanism terminates. In AHT, the injury to the infant is of longer duration and the reflexive adaptive response of hypertension, combined with the shaking stress, causes additional stress in the retina; the two simultaneous stresses from shaking and hypertension cause the blood vessels in the retina to hemorrhage. Therefore, to cause rupture of the blood vessels, both conditions, shaking and hypertension, need to be present to exceed the stress tolerance of the eye.

The article "Modeling Hypertension as a Contributor to Retinal Hemorrhaging from Abusive Head Trauma" was published in 2020. Journal: J Healthc Eng.

## Figures and Tables

**Figure 1:** Circulatory system path of a porcine eye.

**Figure 2:** Diagram of the experimental setup.

**Figure 3:** Perfusion of the porcine retina with dyed Krebs–Ringer solution.

**Figure 4:** RH, the bright green spots, occurring in the porcine eye near splits in the artery.

**Figure 5:** Numerous RHs, the bright green dots, and choroid perfusion, the dull green splotch in the background, seen in the porcine eye.

**Figure 6:** Traced section of the fundus from the porcine eye in DraftSight and exported to COMSOL (r is the retina/choroid domain; b is the blood; and w is the vessel wall; i1 is the inlet, o1, o2, o3 are the outlets; and the POIs are the points of interest).

**Figure 7:** Corresponding stress location points between the FEA model (a) and RH left eye at the initial observation of the locations (b) and the development of the RH (c).

**Table 1:** Material properties used in the FEA model.

	Retina	Blood vessel wall	Blood
Density (kg/m^3^)	1098 [41]	1147 [42]	1057 [42]
Poisson's ratio	0.49 [43]	0.17 [44]	Not applicable
Young's modulus (Pa)	90,000 [43]	192,000 [44]	Not applicable

**Table 2:** Outlet flow velocities.

Outlet	o1	o2	o3
Length (*µ*m)	20	16	18
Velocity (cm/s)	2.13	1.77	1.93

**Table 3:** Settling pressure model POI stress values.

	POI1	POI2	POI3	POI4
von Mises stress (Pa)	184.55	421.95	610.89	791.25
Displacement (*µ*m)	2.41	3.72	5.47	2.71
Volumetric strain	−0.002672	−0.00272	−0.00293	−0.00281

**Table 4:** RH pressure model POI stress values.

	POI1	POI2	POI3	POI4
von Mises stress (Pa)	265.84	598.37	823.69	1082.19
Displacement (*µ*m)	3.37	5.66	8.15	4.13
Volumetric strain	−0.0037	−0.0038	−0.0041	−0.0040

The article "Modeling Hypertension as a Contributor to Retinal Hemorrhaging from Abusive Head Trauma" was published in 2020. Journal: J Healthc Eng.

**Table 5:** Baseline model POI stress values.

	POI1	POI2	POI3	POI4
von Mises stress (Pa)	418.72	908.06	1165.47	1560.17
Displacement (*µ*m)	5.53	8.51	13.2	6.55
Volumetric strain	−0.0057	−0.0059	−0.0063	−0.0062

**Table 6:** TBI mean blood POI values.

	POI1	POI2	POI3	POI4
von Mises stress (Pa)	511.58	1160.99	1300.33	1843.46
Displacement (*µ*m)	7.26	11.2	17.9	9.01
Volumetric strain	−0.0073	−0.0074	−0.0081	−0.0079

**Table 7:** Abusive shaking with TBI blood POI maximum and average values for acceleration.

	POI1		POI2		POI3		POI4	
	Max	Average	Max	Average	Max	Average	Max	Average
von Mises stress (Pa)	578.44	514.30	1361.53	1154.18	1321.47	1285.54	1969.40	1816.51
Displacement (*µ*m)	8.04	7.33	13.33	11.21	23.82	17.80	12.25	9.01
Volumetric strain	−0.0082	−0.0074	−0.0086	−0.0073	−0.0096	−0.0080	−0.0095	−0.0078

**Table 8:** Sans hypertensive shaking model POI maximum and average values for acceleration.

	POI1		POI2		POI3		POI4	
	Max	Average	Max	Average	Max	Average	Max	Average
von Mises stress (Pa)	480.75	420.87	1088.55	919.21	1242.30	1144.93	1784.94	1561.08
Displacement (*µ*m)	6.04	5.56	10.19	8.64	17.69	13.46	8.92	6.74
Volumetric strain	−0.0067	−0.0058	−0.0069	−0.0059	−0.0076	−0.0064	−0.0075	−0.0062

**Table 9:** Stress and displacement change percentage for the POIs and average for the ex vivo RH experimental model and the TBI and abusive shaking TBI models.

		POI1 (%)	POI2 (%)	POI3 (%)	POI4 (%)	
von Mises stress change	Ex vivo RH experimental model	44	42	35	37	Maximum displacement change percentage
	TBI mean blood pressure model	22	28	12	18	
	Nonhypertensive shaking model	15	20	7	14	
	Abusive shaking AHT model	38	*50*	13	26	
Volumetric strain change	Ex vivo RH experimental model	40	41	40	40	
	TBI mean blood pressure model	27	27	29	27	
	Nonhypertensive shaking model	16	17	21	21	
	Abusive shaking AHT model	*45*	*47*	*52*	*54*	

Displacement change	Ex vivo RH experimental model	40	52	49	53	48%
	TBI mean blood pressure model	31	32	36	37	34%
	Nonhypertensive shaking model	9	20	34	36	NA
	Abusive shaking AHT model	*45*	*57*	*81*	*87*	

Values in italics indicate that the computed values exceed the computed experimental increase required to cause RH.

## Data Availability

The experimental and computational data used to support the findings of this study are included within the article. The full set can be found in the author's dissertation (https://ttu-ir.tdl.org/handle/2346/66108) which is cited in the paper.
